The article "Oral Realgar-Indigo Naturalis Formula Treatment for Acute Promyelocytic Leukemia in Children: A Randomized, Control Clinical Trial" was published in 2022. Journal: Evid Based Complement Alternat Med.

# Oral Realgar-Indigo Naturalis Formula Treatment for Acute Promyelocytic Leukemia in Children: A Randomized, Control Clinical Trial

**DOI:** 10.1155/2022/8314176

**Published:** 2022-07-05

**Authors:** Senlin Luo, Jidong Tian, Xiao Sun, Feifeng Wu, Ying Liu, Wuqing Wan, Zhou She, Chuan Wen

**Affiliations:** Department of Pediatrics, The Second Xiangya Hospital, Central South University, Changsha 410011, China

## Abstract

**Objective:**

To analyze the efficacy, safety, and economy of RIF compared with intravenous arsenic trioxide (ATO) for the induction and consolidation therapy of pediatric APL.

**Materials and Methods:**

In this randomized control clinical trial (NCT02200978), children with newly diagnosed APL from June 2013 to December 2017 were randomly divided into RIF and ATO groups. The groups were treated with RIF or ATO in combination with all-trans retinoic acid (ARTA) and conventional chemotherapeutic drugs during induction and consolidation therapy.

**Results:**

Ninteen patients were enrolled, including eight in the RIF group and 11 in the ATO group. After induction therapy, the bone marrow morphologic complete remission (CR) rate, the median time to CR, and molecular remission (promyelocytic leukemia protein (PML)/retinoic acid receptor *α* (RAR*α*) conversion) rates showed no significant differences between patients in the RIF versus ATO groups (100% vs. 100%, *p*=1.000; 22 vs. 24 days, *p*=0.395; 28.5% vs. 54.5%, *p*=0.367, resp.). After consolidation therapy, the molecular remission rate was 100% in both groups. At the end of more than two years of follow-up, the disease-free survival (DFS) rate was 100% in both groups.

**Conclusion:**

Oral RIF can achieve similar efficacy to intravenous ATO for APL in children with good safety, less toxicity, fewer side effects, and fewer inpatient days. Therefore, oral RIF can be used as an alternative to intravenous ATO for the treatment of APL in children.

## 1. Introduction

Acute promyelocytic leukemia (APL), approximately 5–10% of childhood acute myeloid leukemia (AML) cases, is characterized by a chromosome translocation *t*(15; 17), which produced the promyelocytic leukemia protein-retinoic acid receptor *α* (PML-RAR*α*) fusion gene, resulting in the production of PML-RAR*α* oncoprotein [1]. The incidence was 0.06 per 100,000 among those aged below 20 years in the United States during 1975–2008 [2]. The treatment of APL has progressed through three stages: chemotherapy alone, all-trans retinoic acid (ATRA) combined with chemotherapy, and arsenic trioxide (ATO) combined with ATRA and chemotherapy, and the survival rate of patients has continuously improved with each stage. Recent clinical trials have shown that the combination of ATRA and ATO as a first-line treatment for newly diagnosed APL can achieve a high rate of complete remission (CR) and disease-free survival (DFS) [3–7]. The use of ATRA and arsenic for the treatment of APL has been associated with substantial improvements in outcomes, with CR of 90% to 100% of patients in clinical trials and an OS rate more than 95% reported in several trials, and APL is now the most curable subtype of acute myeloid leukemia [8, 9]. The inpatient treatment duration was greatly reduced using the ATO-ATRA regimen [10]; however, ATO must be administered intravenously, which limits any further reduction of inpatient days. Additionally, the intravenous administration of ATO requires the placement of a peripherally inserted central catheter (PICC), which greatly increases the infection rate. Therefore, the potential development of an oral arsenic agent has aroused a great deal of research enthusiasm.

The article "Oral Realgar-Indigo Naturalis Formula Treatment for Acute Promyelocytic Leukemia in Children: A Randomized, Control Clinical Trial" was published in 2022. Journal: Evid Based Complement Alternat Med.

In the 1980s, Chinese scholars developed the Realgar-*Indigo naturalis* formula (RIF, also known as “Fufang Huangdai Pian” in Chinese, ratification number: National Medicine Permit No. Z20090788), which was used for the treatment of APL [11]. In contrast with oral ATO, RIF is a compound preparation containing arsenic, which consists of realgar (also known as XiongHuang, the main component is tetraarsenic tetrasulfide (As_4_S_4_)), *Indigo naturalis* (also known as QingDai, a dark blue powder extracted from the leaves of indigo-bearing plants including *Baphicacanthus cusia* (Ness) Bremek), *Pseudostellariae Radix* (also known as TaiziShen, the dried radix of *Pseudostellaria heterophylla* (Miq.) Pax. (Caryophyllaceae)), and *Salvia miltiorrhiza* (also known as DanShen, the dried radix and rhizome of *Salvia miltiorrhiza* Bunge (Lamiaceae)) [12]. According to traditional Chinese medicine, the pathological basis of APL is that an evil toxin is embedded in the blood, generating blood cancer cells that proliferate endlessly, stagnate in the bone marrow, and infiltrate the viscera and tissue. The nature of the disease is the asthenia of healthy qi and the sthenia of pathogenic factors, which should be treated primarily by removing the poison, expelling the evil, and combining with heat-clearing therapy. Realgar is the monarch drug of RIF, with the main ingredient of tetraarsenic tetrasulfide (As_4_S_4_), which can remove poison, whereas *Indigo naturalis* acts as the minister drug to clear away heat and cool blood, subsequently enhance the effects of realgar. *Pseudostellariae Radix* and *Salvia miltiorrhiza* serve as adjuvant drugs to resolve blood stasis, tonify qi, and activate blood. The compatibility of the four drugs gives them different but complementary roles, which has the effect of expelling evil, clearing away heat, activating blood, and promoting blood generation.

The article "Oral Realgar-Indigo Naturalis Formula Treatment for Acute Promyelocytic Leukemia in Children: A Randomized, Control Clinical Trial" was published in 2022. Journal: Evid Based Complement Alternat Med.

Although studies have examined whether oral RIF can replace intravenous ATO as the first-line component of APL treatment, few systematic reports have been performed in pediatric patients. Additionally, ATO and RIF control in previous studies were mostly examined during the consolidation or maintenance phase. In this randomized controlled trial, a new regimen was designed in which all patients received either ATRA + RIF or ATRA + ATO treatment during both the induction and consolidation phases, and the efficacy, safety, and economy of the two treatment regimens were evaluated and compared to provide a basis for whether oral RIF can replace intravenous ATO in the treatment of APL in children.

## 2. Materials and Methods

### 2.1. Research Subjects

From June 2013 to December 2017, all eligible patients (aged ≤16 years) who were admitted to our department with morphological manifestations of APL, who were positive for *t*(15; 17) on genetic testing, or who were positive for PML-RAR*α* on molecular biological testing were selected for this study. The participant or legal guardian signed the informed consent form. The following exclusion criteria were applied: (1) patients who have coma, convulsion, or paralysis due to intracranial hemorrhage, cerebral thrombosis, or central nervous system leukemia at diagnosis; (2) patients with prolonged QT syndrome during arsenic treatment; (3) patients disagreed with randomized treatment; (4) without a guardian or unable to follow the directions of the medication. The final follow-up time was April 18, 2018.

Patients with APL were risk-stratified according to white blood cell (WBC) and platelet (PLT) counts from peripheral blood testing at admission: low risk: WBC <10 × 10^9^/L and PLT >40 × 10^9^/L; intermediate risk: WBC <10 × 10^9^/L and PLT <40 × 10^9^/L; and high risk: WBC ≥10 × 10^9^/L.

### 2.2. Methods

#### 2.2.1. Study Hypothesis and Groups

This study hypothesized that RIF combined with ATRA would not be inferior to ATO combined with ATRA for the treatment of pediatric APL; oral RIF would reduce inpatient days and medical costs compared with intravenous ATO; and the combination therapy of oral RIF and ATRA would be more convenient for patients than the combination therapy of intravenous ATO and ATRA. Children who met the inclusion criteria were randomly assigned to the RIF and ATRA groups according to the random number table. Patients' families and/or patients provided informed consent. The research followed guidelines of the Declaration of Helsinki and Tokyo for humans and was approved by an ethics committee of clinical investigation. The trial was retrospectively registered in February 2014 at http://www.clinicaltrials.gov as NCT02200978.

The article "Oral Realgar-Indigo Naturalis Formula Treatment for Acute Promyelocytic Leukemia in Children: A Randomized, Control Clinical Trial" was published in 2022. Journal: Evid Based Complement Alternat Med.

#### 2.2.2. Chemotherapy Regimen

The specific chemotherapy regimen applied in this study is shown in Figure 1. During induction and consolidation therapy, the groups were treated with either RIF or ATO combined with ATRA and conventional chemotherapeutic drugs. The varieties and doses of conventional chemotherapeutic drugs depend on risk stratification. For the ATO group, ATO was administered at a dose of 0.16 mg/kg/day (≯10 mg/day) intravenously over 12 hours because prolonging the ATO infusion time can reduce the differentiation and promote the apoptosis of APL cells [13]. Patients assigned to the RIF group received RIF rather than ATO at a dose of 135 mg (half pill)/kg/day (≯30 pills/day) orally three times daily. RIF, also known as Fufang Huangdai Pian in Chinese (GUOYAOZHUNZI Z20090788), was obtained from Tianchang Yifan Pharmaceutical Co., Ltd (Anhui, China), and each tablet (270 mg per pill) contained 30 mg realgar, 125 mg *Indigo naturalis*, 45 mg *Pseudostellariae Radix,* 50 mg *Salvia miltiorrhiza*, and 20 mg garment film (a cover to contain the drug components). The interval between each consolidation course was four weeks, and an intrathecal injection was administered on the first day of each course at the following dose: 2 mg dexamethasone (DXM) + cytarabine (AC) (15 mg for <1 year old, 20 mg for 1–3 years old, and 30 mg for >3 years old). The expression of *PML-RARα* was detected by real-time polymerase chain reaction (RT-PCR) on the first day and at the end of consolidation therapy to determine minimal residual disease (MRD).

#### 2.2.3. Supportive Therapy

At the beginning and during induction therapy, children with WBC >10 × 10^9^/L were treated with oral hydroxyurea (100 mg/kg daily, 2–3 times per day) until WBC <10 × 10^9^/L. When symptoms of induced differentiation syndrome were presented, dexamethasone (0.3–0.5 mg/kg·d) was used until the symptoms disappeared; if the symptoms were serious, ATRA and arsenic were suspended and resumed after symptom improvement. Recurrence was prevented by dexamethasone administration, as appropriate.

Platelet transfusion was performed to increase the platelet count above 30–50 × 10^9^/L (high-risk group must be >50 × 10^9^/L). The transfusion of cold precipitation or fibrinogen preparation was performed to increase blood fibrinogen above 1.5 g/L. If hemoglobin was <60 g/L, the transfusion of suspended red blood cells was performed to improve anemia. Transfusion guidelines were relaxed when weakness was obvious, or the respiratory heart rate was too fast due to anemia. In cases of infection, the infection was actively treated. In cases of neutrophil deficiency, recombinant granulocyte colony-stimulating factor (G-CSF) was used as appropriate. G-CSF was not used during induction therapy.

The article "Oral Realgar-Indigo Naturalis Formula Treatment for Acute Promyelocytic Leukemia in Children: A Randomized, Control Clinical Trial" was published in 2022. Journal: Evid Based Complement Alternat Med.

#### 2.2.4. Safety and Adverse Events

Any serious adverse reactions that occurred during the study were documented. If any adverse event occurred, the investigator determined whether the participant should be withdrawn from the study based on the patient's condition. For serious adverse events, the investigator took necessary measures immediately and reported the event to the ethics committee, with follow-up.

### 2.3. Statistical Analysis

All data were analyzed using SPSS 23.0 software, and the measurement data were described as the mean ± SD or median/interquartile range [M(P25, P75)]. Due to the small sample size, a *t*-test was used to compare variables with a normal distribution, whereas a nonparametric rank-sum test was used to compare variables with a nonnormal distribution. Count data are expressed as the number of cases and percentages, and Fisher's exact test was used for the analysis of these variables. The test level was *α* = 0.05, and *P* < 0.05 was considered significant.

## 3. Results

### 3.1. General Results

Between June 2013 and December 2017, 19 children with newly diagnosed APL were enrolled in this study, and these 19 eligible patients were randomly assigned to receive either RIF and ATRA (*n* = 8) or ATO and ATRA (*n* = 11). The median follow-up times for the RIF and ATO groups were 36.5 months and 32 months, respectively.

### 3.2. Basic Clinical Characteristics

#### 3.2.1. Age at Initial Diagnosis, Gender, and Grouping

Ninteen patients were enrolled in the study, including 10 males and 9 females, with a male-to-female ratio of approximately 1.11 : 1. The median age of the participants was 9 years (range: 1–13 years). Eight patients were placed in the RIF group, including three males and five females, with a median age of 11.5 years (range: 3–13 years), one case in the age group <5 years, six cases in the age group 5–12 years, and one case in the age group ≥13 years. Eleven patients were placed in the ATO group, including four females and seven males, with a median of 6.5 years (range: 1–13 years), two cases in the age group <5 years, eight cases in the age group 5–12 years, and one case in the age group ≥13 years. No significant difference in gender and age composition was observed between the two groups. Of these 19 patients, seven were high-risk patients (1 in the RIF group and 6 in the ATO group), and 12 were low–intermediate-risk (7 in the RIF group and 5 in the ATO group). No significant difference in the risk stratification distribution was observed between the two groups (Table 1).

The article "Oral Realgar-Indigo Naturalis Formula Treatment for Acute Promyelocytic Leukemia in Children: A Randomized, Control Clinical Trial" was published in 2022. Journal: Evid Based Complement Alternat Med.

#### 3.2.2. Molecular Biology

All cases enrolled tested positive for the *PML-RARα* fusion gene before induction therapy, including one case in the RIF group with a positive test for the *FLT-ITD* gene.

### 3.3. Efficacy Analysis

#### 3.3.1. Analysis of Morphological Remission Rate

After induction therapy, all 19 patients (100%) achieved the complete morphological remission of bone marrow. The median times to CR in the RIF and ATO groups were 22 and 24 days, respectively, which was not significantly different (*P* > 0.05; Table 2).

#### 3.3.2. Analysis of the PML-RAR*α* Negative Rate

For *PML-RARα* qualitative test, six of 11 patients in the ATO group tested negative for the *PML-RARα* fusion gene after induction therapy, representing a 54.5% negative rate (6/11). As for RIF group, one patient did not complete the test after induction and consolidation treatment due to poor compliance with medical order, and of the remaining seven patients, two tested negative for *PML-RARα*, representing a 28.5% rate of conversion (2/7). After the consolidation treatment, the conversion rate was 100% in both groups (Table 3).

The quantitative detection of *PML-RARα* was performed, and significant differences were observed in the normalized quantity (NQ) values before and after induction for both the RIF (*P* < 0.05) and ATO groups (*P* < 0.05), indicating that both drug treatments significantly reduced the copy numbers of the *PML-RARα* fusion gene. No significant difference in NQ values was observed between the two groups after induction treatment, suggesting no significant difference between the reductions in fusion gene copy numbers between the RIF and ATO groups (*P* > 0.05). The NQ values decreased to 0 after consolidation therapy for both groups (Table 4).

#### 3.3.3. Survival

All patients completed induction and consolidation therapy, and as of the final study endpoint, the median follow-up time was 32 months (range: 19–52 months) in the ATO group and 36.5 months (range: 4–61 months) in the RIF group, with no significant difference in follow-up time between the two groups (*P*=0.518). By the endpoint of follow-up, all patients survived without morphological or molecular recurrence in the bone marrow, and the DFS rate was 100% for both groups.

### 3.4. Safety Analysis

#### 3.4.1. Adverse Reactions during Induction Therapy

All 19 children experienced varying degrees of adverse reactions during induction therapy. Gastrointestinal reactions manifested as nausea, vomiting, and abdominal pain, whereas respiratory tract infections included acute bronchopneumonia, acute bronchitis, and acute upper respiratory tract infections. The most common adverse reactions during induction in the ATO group were infection, followed by gastrointestinal reactions, whereas the most common adverse reactions during induction in the RIF group were gastrointestinal reactions. No significant differences between the two groups were observed in the total number of adverse events or the distribution of each adverse event during induction therapy (Table 5).

The article "Oral Realgar-Indigo Naturalis Formula Treatment for Acute Promyelocytic Leukemia in Children: A Randomized, Control Clinical Trial" was published in 2022. Journal: Evid Based Complement Alternat Med.

#### 3.4.2. Adverse Reactions during Consolidation Therapy

During consolidation therapy, the most common adverse reactions in the ATO group were infection, gastrointestinal reactions, and headaches. The common adverse reactions in the RIF group were gastrointestinal reactions. The total number of adverse reactions in the ATO group was significantly higher than that in the RIF group (*P* < 0.05). The incidence of headache in the ATO group was significantly higher than that in the RIF group (*P* < 0.05; Table 5).

#### 3.4.3. Analysis of the Effects on the QT Interval

Changes in the QT interval and the QTc interval before induction therapy and after the end of induction and consolidation therapy were compared between the two groups. The results showed significant differences in the QT and QTc interval values before and after treatment in the ATO group (*P* < 0.05), whereas no significant differences were observed before and after treatment in the RIF group, which indicated that ATO treatment affected the QT and QTc intervals of patients more than the RIF treatment (Table 6).

### 3.5. Economic Analysis

When analyzing the inpatient days from the beginning of induction to the end of consolidation therapy, the mean number of inpatient days was significantly reduced in the RIF group compared with that in the ATO group (*P* < 0.05; Table 7).

## 4. Discussion

APL is a unique subtype of AML that accounts for 10%–34% of acute leukemia in children [14–16]. The treatment of APL has gone through three stages: traditional chemotherapy, ATRA combined with chemotherapy, and ATRA combined with ATO and chemotherapy. During the early treatment stages using simple chemotherapy, the risk of death was high due to the poor effects of drug therapy [17]. The mechanism of ATRA treatment is to restore the activities of the RAR*α* and PML genes by targeting the degradation of the PML-RAR*α* oncoprotein [18], and the CR rate and long-term survival rate associated with treatment consisting of ATRA combined with chemotherapy can reach approximately 90% and 85%, respectively [19, 20]. However, some patients can develop more severe myelosuppression or secondary forms of other AMLs during treatment with this regimen [21, 22]. In addition, if ATRA resistance occurs, the relapse rate increases among high-risk patients [23]. ATO, a major component of Chinese medicine preparation arsenic, can shorten the treatment time, reduce the occurrence of myelosuppression, and reduce the relapse rate by inducing promyelocyte differentiation and apoptosis and PML-RAR*α* fusion protein degradation [24, 25]. When treated with ATO combined with ATRA and chemotherapy, the cure rate can reach approximately 95% [26], making APL a curable disease [27–29].

The article "Oral Realgar-Indigo Naturalis Formula Treatment for Acute Promyelocytic Leukemia in Children: A Randomized, Control Clinical Trial" was published in 2022. Journal: Evid Based Complement Alternat Med.

The efficacy of RIF for the treatment of APL has been gradually confirmed in clinical trials. In patients with newly diagnosed APL, the outcome of Phase 2 clinical trials of RIF for APL treatment by the Institute of Hematology of the Chinese Academy of Medical Sciences showed that the CR rate of RIF treatment was as high as 96.7%–100% [30]. For patients with refractory APL, Liu et al. reported an overall sustained CR rate of 90.32% (28/31) for RIF treatment [31]. Several studies have shown that differences in the CR and DFS rates between RIF and ATO were not significant, suggesting that the RIF combined with ATRA regimen is at least not inferior to the standard ATO combined with ATRA regimen [32–34]. Fewer studies have examined RIF treatment in children. Zhu et al. used RIF combined with ATRA for induction chemotherapy in nine nonhigh-risk children, all of whom achieved CR at a median time of 30 days, with two-year predicted EFS and OS values of 100% [35].

In our study, both groups achieved CR after induction therapy, and no significant differences were identified in CR rate, time to reach CR, or the rate of PML-RAR*α* conversion after treatment between the RIF and ATO groups. The DFS rate was 100% in both groups at the final follow-up endpoint, a result that further validates the effectiveness of both arsenic agents, suggesting that oral RIF is not inferior to intravenous ATO for the treatment of pediatric APL.

The efficacy of RIF in APL is not inferior to that of ATO due to its unique mechanism. As4S4, which is the main active ingredient of realgar in RIF, can induce apoptosis in HL-60 and NB4-R1 cells [36–39]. Wang and Liu et al. demonstrated that As4S4 could significantly induce the degradation of the PML-RAR*α* oncoprotein in mouse models and in vitro experiments. Indirubin, the main active component of indigo naturalis, significantly inhibits the cell cycle, and tanshinone, the main active component of *Salvia miltiorrhiza*, significantly promotes the expression of cell differentiation genes. In addition, indirubin and tanshinone can intensify the expression of aquaglyceroporin 9, which facilitate the transportation of As4S4 into APL cells, ultimately enhancing As4S4-mediated PML-RAR*α* degradation and therapeutic efficacy [12, 31]. Therefore, RIF differs from ATO because its mechanism of action, in addition to inducing the cleavage of the PML-RAR*α* oncoprotein, also hits multiple targets. In addition, interactions between each component in RIF promotes the activities of the other components, enhancing the anti-APL effects of arsenic. Salvia miltiorrhiza and Pseudostellariae Radix also promote the restoration of normal hematopoietic function, prevent disseminated intravascular coagulation (DIC), bleeding, and infection, and ultimately enhance the therapeutic efficacy and reduce adverse effects of RIF [40].

The article "Oral Realgar-Indigo Naturalis Formula Treatment for Acute Promyelocytic Leukemia in Children: A Randomized, Control Clinical Trial" was published in 2022. Journal: Evid Based Complement Alternat Med.

The long-term use of arsenic agents can have toxic side effects. Chinese clinical trials and Zhu et al. reported mild adverse reactions in patients with APL who were treated with RIF combined with ATRA, although the differences were not significant when comparing adverse reactions between the RIF and ATO groups [30–32, 34]. The patients in our study experienced varying degrees of adverse reactions during treatment, and the total number of adverse reactions was lower in the RIF group than that in the ATO group during consolidation therapy. During treatment, the primary adverse reaction in the ATO group was infection, which was likely associated with drug-induced myelosuppression and the PICC line insertion. In contrast, the primary adverse reaction in the RIF group was gastrointestinal discomfort, which was likely associated with oral administration-induced gastrointestinal reactions. The number of headache events was higher in the ATO group than in the RIF group during consolidation therapy, and headache may be caused by ATRA and/or arsenic agents, the specific mechanism of which requires additional study. The interaction between the various components of RIF promoted each other and enhanced the anti-APL effect of arsenic, allowing RIF to be used at a lower therapeutic dose of arsenic, which reduced toxicity. Moreover, Salvia miltiorrhiza and Pseudostellariae Radix can protect the functions of the heart, liver, kidney, and other organs [40], reducing toxic side effects.

The prolongation of QT intervals occurs in some patients during arsenic administration; therefore, this study monitored the QT and QTc intervals through regular electrocardiography. The results showed that the QT and QTc intervals were more affected in the ATO group than in the RIF group. QT interval prolongation is a common side effect of ATO [41–44], and 7.5% of APL patients treated with ATO in the study reported by Abaza et al. experienced QT interval prolongation [45]. In addition, the GIMEMA-SAL-AMLSG APL0406 trial reported QTc interval prolongation in 16% of patients in the ATRA + ATO group [46]. However, prolonged QTc intervals and severe arrhythmias have not been reported after oral RIF administration in recent trials using RIF combined with ATRA as first-line therapy [32, 47–49]. Intravenous ATO is more likely to prolong the QT or QTc interval than oral RIF, which may be related to the rapid increase in the blood arsenic concentration and the higher accumulation of arsenic in cardiac tissues due to intravenous administration. The difference may also be related to the rarer occurrence of electrolyte disturbances, such as hypokalemia and hypomagnesemia, during RIF treatment.

The article "Oral Realgar-Indigo Naturalis Formula Treatment for Acute Promyelocytic Leukemia in Children: A Randomized, Control Clinical Trial" was published in 2022. Journal: Evid Based Complement Alternat Med.

In this study, the inpatient days for induction and consolidation treatment were significantly reduced in the RIF group compared with the ATRA group, and the costs of hospitalization decreased accordingly, which could reduce the financial burden for patients. The total medical costs reported for the home treatment model of RIF + ATRA was significantly lower than the costs for the intravenous ATO group [50, 51].

In conclusion, this clinical study showed that the RIF and ATO groups achieved similar CR and DFS rates. The adverse reactions of the RIF group were not significantly different from those of the ATO group during treatment, but the incidence of infections was reduced. However, the inpatient days in the RIF group were significantly reduced compared with those in the ATO group, reducing the economic burden of patients and the discomfort caused by inpatient infusions, suggesting that RIF can improve patients' quality of life with shorter hospital stays and lower costs while achieving similarly high remission rates and survival outcomes.

## 5. Conclusions

Oral RIF can achieve similar efficacy to intravenous ATO during the induction and consolidation phases of APL in children with good safety, less toxicity, fewer side effects, and fewer inpatient days. Therefore, oral RIF can be used as an alternative to intravenous ATO for the treatment of APL in children.

## Figures and Tables

**Figure 1:** Chemotherapy regimen. RIF: realgar-*indigo naturalis* formula; ATO: arsenic trioxide; ATRA: all-trans retinoic acid; MA: mitoxantrone; AC: cytarabine; CR: hematologic complete remission; MRD: minimal residual disease; IT: intrathecal injection.

**Table 1:** Baseline characteristics.

	RIF group (*n* = 8)	ATO (*n* = 11)	*t-*value	*p*-value
Sex (*n*)				
Male	3	7		0.375^*∗*^
Female	5	4		
Median age (years)	10.12 ± 3.2	7.36 ± 3.6	−1.693	0.100
Age group (*n*)				
＜5 years	1	2		
5–12 years	6	8		
≥13 years	1	1		
Sanz risk (*n*)				
Low–intermediate	6	5		0.310^#^
High	2	6		

^#^Nonparametric test. ^*∗*^Fisher's exact test. RIF: realgar-indigo naturalis formula; ATO: arsenic trioxide.

The article "Oral Realgar-Indigo Naturalis Formula Treatment for Acute Promyelocytic Leukemia in Children: A Randomized, Control Clinical Trial" was published in 2022. Journal: Evid Based Complement Alternat Med.

**Table 2:** Remission rate after induction therapy.

	RIF	ATO	*p*-value
CR rate	100% (8/8)	100% (11/11)	1.000^#^
Days to CR [M (P_25_, P_75)_]	22 (20, 24)	24 (22, 29.5)	0.395^#^

^#^Nonparametric test. RIF: realgar-indigo naturalis formula; ATO: arsenic trioxide; CR: complete remission; M: median; P25: 25th percentile; P75: 75th percentile.

**Table 3:** Qualitative test results of *PML-RARα* before and after induction therapy.

		Before (*n*)		After (*n*)		Negative rate (%)	*p*-value
		Positive	Negative	Positive	Negative		
*PML-RARα* qualitative test	RIF group	8	0	5	2	28.5%	0.367^*∗*^
	ATO group	11	0	5	6	54.5%	

^*∗*^Fisher's exact test. RIF: realgar-indigo naturalis formula; ATO: arsenic trioxide; PML: promyelocytic leukemia protein; RAR*α*: retinoic acid receptor *α*.

**Table 4:** Quantitative test results of *PML-RARα* before and after induction therapy.

*PML-RARα* (NQ value)	RIF group (*n* = 7)	ATO group (*n* = 11)	*p*-value
Before [M (P_25_, P_75_)]	0.262(0.209, 0.786)	0.235(0.145, 0.612)	0.633^#^
After [M (P_25_, P_75_)]	0.008(0.000, 0.072)	0.000(0.000, 0.004)	0.179^#^
*p* value	0.000^#^	0.000^#^	

^#^ Nonparametric test; RIF: realgar-indigo naturalis formula; ATO: arsenic trioxide; NQ: normalized quantity; M: median; P25: 25th percentile; P75: 75th percentile.

**Table 5:** Incidence of adverse reactions following two courses of treatment (*n* (%)).

	Induction phase			Consolidation phase		
	ATO (*n* = 11)	RIF (*n* = 8)	*p*-value	ATO (*n* = 11)	RIF (*n* = 8)	*p*-value
Respiratory infection	8 (72.70%)	4 (50.00%)	0.297^*∗*^	7 (63.63%)	2 (25%)	0.115^*∗*^
Gastrointestinal reaction	7 (63.63%)	7 (87.50%)	0.267^*∗*^	7 (63.63%)	5 (62.5%)	0.663^*∗*^
Rash	1 (9.09%)	1 (12.50%)	0.678^*∗*^	1 (9.09%)	0 (0)	0.111^*∗*^
Headache	4 (36.36%)	4 (50.00%)	0.449^*∗*^	7 (63.63%)	1 (12.5%)	0.037^*∗*^
Sepsis	1 (9.09%)	0 (0)	0.579^*∗*^	1 (9.09%)	0 (0)	0.579^*∗*^
Hepatic toxicity	0 (0)	3 (37.50%)	0.058^*∗*^	1 (9.09%)	1 (12.5%)	0.678^*∗*^
Fundal hemorrhage	0 (0)	1 (12.50%)	0.421^*∗*^	1 (9.09%)	0 (0)	0.579^*∗*^
Arthralgia	1 (9.09%)	1 (12.50%)	0.678^*∗*^	0 (0)	0 (0)	—
DIC	1 (9.09%)	1 (12.50%)	0.678^*∗*^	0 (0)	0 (0)	—
Cardiac toxicity	0 (0)	0 (0)	—	1 (9.09%)	0 (0)	0.579^*∗*^
	23	22	0.556^*∗*^	26	9	0.019^*∗*^

^*∗*^Fisher's exact test; RIF: realgar-indigo naturalis formula; ATO: arsenic trioxide.

**Table 6:** QT and QTc intervals (millisecond, $\bar{x}\pm s$).

	ATO group				RIF group			
	Before therapy	After therapy	*t-*value	*p*-value	Before therapy	After therapy	*t-*value	*p*-value
QT	321.64 ± 46.843	381.18 ± 39.133	−3.236	0.004	362 ± 44.246	398.286 ± 56.467	−1.397	0.186
QTc	433.91 ± 29.218	465.00 ± 27.796	−2.557	0.019	450 ± 29.277	474.571 ± 33.075	−1.527	0.151

RIF: realgar-*indigo naturalis* formula; ATO: arsenic trioxide.

The article "Oral Realgar-Indigo Naturalis Formula Treatment for Acute Promyelocytic Leukemia in Children: A Randomized, Control Clinical Trial" was published in 2022. Journal: Evid Based Complement Alternat Med.

**Table 7:** Total inpatient days for induction and consolidation therapy.

	RIF	ATO	*t-*value	*p*-value
Total inpatient days	50.50 ± 12.98	81.64 ± 8.68	6.282	0.000

RIF: realgar-*indigo naturalis* formula; ATO: arsenic trioxide.

## Data Availability

The data used to support the findings of this study are available from the corresponding author upon request.
